# RAGE Regulating Vascular Remodeling in Diabetes by Regulating Mitochondrial Dynamics with JAK2/STAT3 Pathway

**DOI:** 10.1155/2022/2685648

**Published:** 2022-04-22

**Authors:** Shengjia Sun, Qiying Chen, Bangwei Wu, Qingyu Huang, Alimujiang Maimaitijiang

**Affiliations:** Department of Cardiology, Huashan Hospital Fudan University, No.12 Urumqi Middle Road, Shanghai 200040, China

## Abstract

In this research, we will explore the role and modulation of mitochondrial dynamics in diabetes vascular remodeling. Only a few cell types express the pattern recognition receptor, also known as the AGE receptor (RAGE). However, it is triggered in almost all of the cells that have been investigated thus far by events that are known to cause inflammation. Here, Type 2 diabetes was studied in both cellular and animal models. Elevated Receptor for advanced glycation end products (RAGE), phosphorylated JAK2 (p-JAK2), phosphorylated STAT3 (p-STAT3), transient receptor potential ion channels (TRPM), and phosphorylated dynamin-related protein 1 (p-DRP1) were observed in the context of diabetes. In addition, we found that inhibition of RAGE was followed by a remarkable decrease in the expression of the above proteins. It has also been demonstrated by western blotting and immunofluorescence results in vivo and in vitro. Suppressing STAT3 and DRP1 phosphorylation produced effects similar to those of RAGE inhibition on the proliferation, cell cycle, migration, invasion, and expression of TRPM in VSMCs and vascular tissues obtained from diabetic animals. These findings indicate that RAGE regulates vascular remodeling via mitochondrial dynamics through modulating the JAK2/STAT3 axis in diabetes. The findings could be crucial in gaining a better understanding of diabetes-related vascular remodeling. It also contributes to a better cytopathological understanding of diabetic vascular disease and provides a theoretical foundation for novel targets that aid in the prevention and treatment of diabetes-related cardiovascular problems.

## 1. Introduction

The RAGE (receptor for AGEs) type I transmembrane receptor is a relatively new member of the immunoglobulin superfamily. RAGE (also known as AGER) is found on chromosome 6 in the gene-dense major histocompatibility class III region, which includes several genes implicated in inflammatory and immunological responses, including TNF (also known as TNF) and various complement components. The vascular consequences of diabetes are caused by the abnormal remodeling of blood arteries caused by advanced glycation end products (AGEs) and their signal transduction receptors (RAGEs) (AGEs-RAGE axis). Despite considerable and in-depth basic and clinical research, cardio-cerebrovascular disorders continue to be the primary cause of death in humans around the world [1]. As a condition with an equal risk of coronary artery disease, diabetes can considerably raise the risk of cardio-cerebrovascular disorders, with ischemic cardio-cerebrovascular consequences accounting for three-quarters of all diabetes-related deaths [2]. From vitro experiments to pathophysiological analysis, including epidemiological studies, numerous studies have confirmed that the pathophysiological response mediated by AGEs and RAGEs in vascular remodeling in diabetes is critical in the onset and progression of ischemic vascular complications. The oxidative stress response, cell multiplication, migration, and phenotypic alteration of vascular smooth muscle cells (VSMCs) induced by the AGEs-RAGE axis, as well as extracellular matrix creation, are all key pathogenic bases for diabetic vascular remodeling [3]. However, until now, clinically, there is still a lack of effective interventions to block the effect of RAGE. Also, to exact mechanism of the RAGE effect on VSMC is still unclear [4].

Mitochondria are mammalian cells' principal source of energy, regulating cell signaling, proliferation, reactive oxygen species (ROS), and apoptosis [5]. It is highly dynamic organelles, maintain a balanced network of mitochondria through continuous fusion and division. This dynamic process is called mitochondrial dynamics. This process consists of a series of reactions regulated by dynein's bound to GTPase [6], mainly the proteins bound to the mitochondrial fusion (mitofusin1 (Mfn1), mitofusin2 (Mfn2)) and the protein bound to the mitochondrial dynamin-related protein (Drp1). Carboxymethyllysine-bound albumin (CML-BSA) is the major component of EFAs. Studies have confirmed that CML-BSA intervention can lead to decreased mitochondrial membrane potential and ATP synthesis, upregulation of ROS synthesis and lipid peroxidation, increased levels of Drp1, and an increase in the mitochondrial division. It confirms that AGEs can interfere with mitochondrial function and kinetic changes [7]. In a previous study, we discovered that using the specific Drp1 inhibitor Mdivi-1 (Mitochondrial division inhibitor 1) can inhibit the hyperproliferation of VSMCs induced by high glucose conditions, promote mitochondrial fusion, and reduce ROS production, potentially counteracting the damage caused by oxidative stress in high glucose conditions [8]. Through recent preliminary experiments, we have found that CML-BSA can also promote VSMC proliferation and mitochondrial division, dramatically increase the level of Drp1, and down-regulate Mfn2 expression; these effects of CML-BSA were effectively reversed by Mdivi-1. Additionally, we also found that Mdivi-1 significantly down-regulated the level of RAGE expression. It can effectively oppose the promoter effect of AGEs on RAGE expression. This suggests that the mitochondrial fusion and division activities of VSMCs can be used as intervention targets to regulate RAGE expression and antagonize diabetes-related vascular remodeling.

The JAK/STAT (Janus kinase/signal transducers and activators of transcription) axis transmits chemical signals (interferons, interleukins, growth factors, etc.) from the outside of the cell to the nucleus, triggering DNA transcription and expression of genes associated with immunity, cell multiplication, differentiation, apoptosis, and tumorigenesis. The JAK family, in mammals, consists of JAK1-3 and Tyk2. While STAT1-4, STAT5a, STAT5b, and STAT6 are among the seven members of the STAT family identified so far [9]. The JAK/STAT axis had previously been studied for its role in carcinogenesis and metastasis. In recent years, attention has focused to its role in VSMC proliferation, migration, and phenotypic transition regulation. For example, JAK2/STAT3 may participate in modulating phenotypic transformation of VSMCs in the middle aorta of hypertensive rats [10]. PA2 (proanthocyanidin A2) can inhibit the proliferation of VSMCs induced by PDGF via the JAK2/STAT3 signaling pathway [11]. We discovered through preliminary experiments that CML-BSA can significantly up-regulate phosphorylation levels of JAK2 and STAT3 while promoting VSMC proliferation and mitochondrial division, and the intervention of Mdivi-1 can effectively reverse these effects. This suggested that regulation of the JAK2/STAT3 signaling pathway on VSMC proliferation may be affected by changes in mitochondrial dynamics. However, the specific mechanisms by which changes in the mitochondrial dynamics of VSMCs are affected by the JAK2/STAT3 signaling pathway are unknown. Furthermore, whether this signaling pathway is a key regulatory factor involved in diabetic vascular remodeling is not explained.

In order to answer this question, this study used C57BL/6 mice to model type 2 diabetes and aortic VSMCs of mice to conduct cellular experiments. Our main objectives are summarized as follows:

- To observe at the cellular level and in vivo, whether the level of RAGE expression in smooth muscle cells affects mitochondrial dynamics and the JAK2/STAT3 axis
- To study the effects of the JAK2/STAT3 axis and mitochondrial dynamics on VSMC proliferation, migration, and phenotypic transformation

The remainder of the research study is organized in the following manner. The material, methods, and instruments used in this investigation will be explained in the next section. After then, the findings of this study will be presented. Finally, towards the end of this study report, there is a discussion of the findings and some concluding thoughts.

## 2. Material and Methods

In this section, we will go over how the diabetic mouse model was created, as well as the many stages and tests performed on the study subject. The explanation is simple to understand.

### 2.1. Establishment of the Diabetic Mouse Model

Wild type C57BL/6J mice (about 3 weeks of age; SLAC Laboratory Animal Co. Ltd., Shanghai, China) were housed in a room respecting the following conditions: light/dark cycle of 12/12 hours, 60% humidity, and temperature of 23 ± 2°C, with water and chow available ad libitum. After acclimatization of 14 days, the distribution of the mice into different groups (each with 30 mice) was made at random as follows: control, DM, T2DM, the T2DM + DMSO, T2DM + Mdivi (50 mg/kg, i.p.; twice per week), T2DM + stattic group (10 mg/kg; i.p.; three times per week), T2DM + siNC and T2DM + siRAGE group. Induction of diabetes: streptozotocin (STZ), (intraperitoneal dose of 60 mg/kg/d that was dissolved in 0.1 mol/L of citrate buffer, pH 4.5; Sigma-Aldrich) over a period of 5 days. Mice were declared diabetic if their blood glucose level was ≥16.7 mmol/L 8 days after STZ administration. In the siRAGE group, the T2DM mice were administered with RAGE siRNA (siRAGE) (5 *μ*g), which was preliminarily prepared by mixing transfection solution (40 *μ*l) (NANOPARTICLE, Altogen Biosystems, Las Vegas, NV, USA) with 5% glucose (w/v), in a final volume of 100 *μ*l. A similar protocol with NC siRNA was performed. One month after the first injection, the diabetic mice were reinjected with the equivalent concentration of the siNC or siRAGE. Weight and blood sugar gains were taken weekly after STZ induction. This study was ratified by the Animal Ethical Committee of Huashan Hospital Fudan University, China, and the research work was conducted in the School of Medicine, Fudan University. The National Institutes of Health (NIH) recommendations were followed during mouse experiments. Isoflurane anesthesia (5%) was administered to the animals prior to cervical dislocation.

### 2.2. Histological Analysis

Aorta samples isolated from mice were taken and fixed in formaldehyde (4%) before paraffin-embedding. Then, 5 *μ*m thick cross-sections were prepared. It was followed by hematoxylin and eosin (HE) staining and the subsequent photographing with the Nikon brand optical microscope at the original magnification of 200X.

### 2.3. Cell Culture and Processing

MOVAS, a mouse VSMC line supplied by ATCC, was grown at 37°C in DMEM (Gibco Invitrogen) (25 mmol/L D-glucose, 200 *μ*g/mL geneticin, 10% fetal bovine serum) in a 5% CO2 incubator. They were first cultivated under normoglycemic conditions (5.5 mmol/L glucose) for a period of 12 hours before exposure to hyperglycemic conditions (33 mmol/L glucose) at various time intervals. Cells after 3–8 passages were used in the rest of the experiments. For experiments, aliquots of 5*∗*106 cells were treated on the following day with 6 *μ*M CML-BSA (Toronto, Canada) for 24H. 25 *μ*M Mdivi-1 (sigma Chemical, St. Louis, MO) for specific inhibition of DRP1 for 48H and 20 *μ*M stattic (MCE Chemical, USA) were added for specific inhibition of STAT3 for 24H.

### 2.4. Transfection of siRNA into VSMCs Cells

The transfection of RAGE-RNAi lentiviruses against RAGE (Shanghai Genechem Co. Ltd.) into VSMCS cells was performed with Lipofectamine (Invitrogen) following the manufacturer's recommendations. Target siRNA sequence was 5′-AGTCCGTGTCTACCAGATT-3′. While the contrast insertion sequence was 5′-TTCTCCGAACGTGTCACGT-3′. A scrambled probe functioned as the control. Following transfection, cells were immersed in a normal medium containing glucose for 24 hours of cultivation. Thereafter, the normal medium was replaced with a hyperglycemic medium for an additional 24 hours of cell culture. The cells obtained were recovered for subsequent analyses.

### 2.5. Analysis of Cell Proliferation

Following the methodology described in a previous paper, the MTT test was performed to assess cell viability after various treatments. The formazan produced upon incubation with 0.5 mg MTT reagent was then dissolved in dimethyl sulfoxide (DMSO). The optical density was measured colorimetrically at 490–630 nm with the use of a microplate reader.

### 2.6. Cell Cycle Analysis

For the analysis of cell cycle phases, cells were collected from culture plates using 0.05% trypsin/EDTA. After centrifugation, they were immobilized with well-chilled 70% ethanol (2 mL) with vigorous shaking. After standing on ice for 1 hour (h), cells were stored at 4°C for ≥48 h to remove the fragmented DNA from apoptotic cells. The fixed cells were subjected to two washes with PBS, followed by incubation in the dark in PBS in the presence of RNase A (50 ng/mL) and PI (1 mL, 50 mg/mL) for 3 h at 4°C. Collection of fluorescence data was done in the FL3 channel at a linear scale of 10,000 cells/sample. A Cytoflex flow cytometer (Beckman Coulter Ltd., Brea, CA, USA) was employed for sample analysis and the percentage of cells in different cell cycle phases was measured.

### 2.7. Wound Healing Test

For this purpose, approximately 200,000 cells/well were inoculated into 24-well plates for 24 hours without food. Subsequently, the replacement of the culture medium with a medium containing 10% FBS was carried out. A plastic tip was used to induce injury by passage through the monolayer cells. The wound induction time was considered the initial time (0 h). The photographs were taken after 48 hours with a microscope coupled to a digital camera to assess wound closure. The regions occupied by the migrating cells were measured using ImageJ 1.48v software and expressed as a percentage. All of the trials were carried out three times.

### 2.8. Transwell Assay

After starving the cells in a serum-free medium, a cell suspension was inoculated into each well of the transwell chamber (8 *μ*m pore size, Corning, New York, USA) pre-coated with a membrane of Matrigel (BD Biosciences, San Jose, CA, United States). RPMI medium mixed with 10% FBS was placed in the basolateral chamber. The chambers were incubated for a period of 24 hours in a humidified incubator (37°C, 5% CO2) and the cells which had not crossed the membrane and remained on the apical chamber were cleaned with Q-tips. Subsequently, methanol was used to fix the cells on the underside of the upper chamber. It was followed by 10 min of crystal violet (2%) staining. The cells which had crossed the membrane were enumerated microscopically in five random visual fields. The experiments were done in a triplet.

### 2.9. ROS Detection by Flow Cytometry

The detection of ROS in the different groups of cells was performed by flow cytometry. The DCFH-DA probe was used for the detection of intracellular ROS under excitation at a wavelength of 488 nm. The fluorescence emission was measured in the FL1 533 area. The measurements were taken around 30 minutes after the cultivated cells had been incubated in DMEM without FBS at 37°C. The BD Accuri C6 flow cytometer was utilized to detect the cells.

### 2.10. Mitochondrial Membrane Potential (MMP or ΔΨm) Assay

The cells in each group were subjected to 30 min of cultivation with JC-1 reagent (1 *μ*g/mL) at 37°C in a culture medium. After which they were processed for PBS washing again and subsequent photographing with the use of a fluorescence microscope (Leica TCS SP5, Leica Co. Ltd). The red/green fluorescence intensity ratio was then computed.

### 2.11. Immunofluorescence

The measurement of TRPM, *α*-SMA, CD31, and VEGF expression was made using the immunofluorescence method. Following their fixation and permeabilization, aortic tissue slices or VSMCs collected from different groups were cultivated at 4°C with antibodies (dilution: 1 : 500) against TRPM, *α*-SMA, CD31, and VEGF overnight. TRPM, *α*-SMA, CD31, and VEGF were labeled with goat anti-mouse antibodies. After this, the sections were counterstained with DAPI (blue). Finally, using a confocal laser scanning microscope, fluorescence images were captured (Leica TCS SP5, Leica Co. Ltd).

### 2.12. Western Blot

The homogenization of VSMCS cells and isolated aortic tissues were performed by immersing them in RIPA lysis buffer + protease and phosphatase inhibitors (Roche). After being quantified with Thermo Fisher Scientific's BCA Protein Assay Reagent, identical aliquots of total protein (30–60 g) were electrophoresed on SDS-PAGE (8 percent or 10%) before being transferred to PVDF membranes. After indoor incubation in blocking buffer containing NaCl (150 mmol/L), skim milk (5%), Tris-HCl (20 mmol/L) Tween-20 (0.05%, pH 7.6) for a period of 2 hours, the membranes were subjected to overnight cultivation (4°C) with first antibodies directed against GAPDH, JAK2, p-JAK2, STAT3, p-STAT3, Mfn2, Drp1, p-Drp1, CD31, and VEGF-A (dilution 1 : 1000; all from Cell Signaling Technology Inc) in 5% BSA. After three washes of 10 minutes each in saline plus Tween-20 (1x TBST), they were cultivated with a secondary antibody (1 : 1000; Cell Signaling Technology) for a period of 2 hours, followed by chemiluminescence visualization. ImageJ software was used for the densitometric analysis of immunoreactive bands.

### 2.13. Statistical Processing

The experiments were repeatedly determined three times and the data were denoted as mean ± SD. The method used for inter-group comparison was one-way ANOVA and the *p*-value cutoff was 0.05. The software adopted for analysis was GraphPad Prism (GraphPad Prism Software Inc., San Diego, CA, USA).

## 3. Results

The results of different experiments done in this research are as follow;

### 3.1. RAGE Regulates Mitochondrial Dynamics and JAK2/STAT3 Pathway in Diabetes

To specify the regulatory effect of the AGE-RAGE signaling pathway in vascular remodeling linked to the context of diabetes, we first carried out different treatments of VSMCs cells. Analysis of the expression of important proteins was done using the western blot method. It turned out that after treatment of VSMCs cells with CML-BSA, RAGE and the phosphorylated forms of the STAT3 (p-STAT3) and JAK2 (p-JAK2) proteins were upregulated while the expression levels of JAK2 and STAT3 had remained almost unchanged (Figure 1(a)). There was also an increase in the expression of the phosphorylated Drp1 (p-Drp1) protein, but MFN2 expression was significantly reduced (Figure 1(a)). The suppression of the RAGE protein was done with siRNAs to confirm the probable control of the aforesaid proteins by RAGE. As RAGE was silenced, the effect of CML-BSA was suppressed, as seen by a drop in p-STAT3, p-JAK2, and p-DRP1 levels, as well as an increase in MFN2, when compared to the CML-BSA and CML-BSA + siNC groups (Figure 1(a)). The analysis of the immunofluorescence with TRPM showed that the expression of this protein was induced by the treatment of CML-BSA versus the control group, but such effect was suppressed by the inhibitory action of RAGE (Figure 1(b)). Second, we established an animal model of type 2 diabetes by STZ injection. It was observed that p-STAT3, p-JAK2, and p-DRP1 were elevated in vascular tissues of diabetic mice versus non-diabetic ones (Figure 2). In addition, the expression of MFN2 decreased compared to the control group (Figure 2). Similar to in vitro experiments, inhibition of RAGE was accompanied by a significant abrogation of the effect of STZ on the expression of p-STAT3, p-JAK2, p-DRP1, and MFN2 (Figure 2). These experiments showed that RAGE could control the regulation of vascular remodeling by activating the JAK2/STAT3 pathway.

### 3.2. RAGE-Mediated Activation of JAK2/STAT3 Axis Regulates VSMC Proliferation, Cell Cycle, Migration, And Invasiveness

To analyze whether the activating effect of RAGE on the JAK2/STAT3 signaling pathway is involved in vascular remodeling, several treatments with mitochondrial division inhibitor 1 (Mdivi-1), STAT3 inhibitor (stattic), and the RAGE siRNAs were performed and their effect on the expression of the above-mentioned proteins was verified by western blotting. Treatment with Mdivi-1 effectively inhibited p-DRP1 expression. While stattic effected hindered p-STAT3 expression (Figure 3(a)). In addition, Mdivi-1 allowed the reversal of the effect of CML-BSA on the expression of MFN2, p-STAT3, and p-JAK2 (Figure 3(a)). Similar observations were made with stattic treatment and RAGE siRNAs (siRAGE). In the cell model, we found that treatment with CML-BSA led to the increase of cell proliferation; treatments with Mdivi-1, stattic, or siRAGE made it possible to reverse the influence of CML-BSA on VSMC proliferation (Figure 3(b)). Afterwards, we measured the effect of the different treatments on the cell cycle by flow cytometry. As shown in Figure 4(a), treatment with CML-BSA led to a rise in the number of G2-phase cells. However, treatments with Mdivi-1, stattic, or siRAGE all blocked this trend. No significant change was recorded in the percentage of G1-and S-phase cells. This indicated that Mdivi-1, stattic, or siRAGE reversed the activation effect of CML-BSA on cell proliferation by unblocking CML-BSA-induced cell cycle arrest at the G2 phase. The wound-healing test and Transwell assay showed that Mdivi-1, stattic, and siRAGE all reversed the induction effect of CML-BSA on cell migration (Figure 4(b)) and invasiveness (Figure 4(c)).

### 3.3. RAGE-Mediated Activation of JAK2/STAT3 Axis Regulates ROS and Mitochondrial Dynamics of VSMCs in Diabetes

To determine RAGE regulates ROS, the determination of ROS by flow cytometry was performed. As shown in Figure 5(a), treatment with CML-BSA resulted in increased ROS in VSMCs compared to normal cells. In addition, after treatment with Mdivi-1, stattic, and siRAGE, the level of ROS decreased compared to cells treated with CML-BSA (Figure 5(a)).

In the analysis of protein expression of markers of vascular remodeling, we noted an increase in the expression of *α*-SMA and CD31 following treatment of VSMCs cells with CML-BSA; this effect was inhibited by treatments with Mdivi-1, stattic, and siRAGE (Figure 5(b)). In addition, we noted that Mdivi-1, stattic, and siRAGE all inhibited the expression of VEGF-A induced by CML-BSA (Figure 5(b)). In addition, immunofluorescence of TRPM showed that induction of this protein by CML-BSA was abrogated by treatment with Mdivi-1, stattic, and siRAGE (Figure 6). More notably, an MMP (m) assay using the JC-1 staining method revealed considerable depolarization of the MMP in the CML-BSA induction group, although this effect was blocked by Mdivi-1, stattic, and siRAGE therapy (Figure 7(a)). In the control group, JC-1 emitted red fluorescence, but after CML-BSA induction, JC-1 emitted green fluorescence with little red fluorescence; however, treatment with Mdivi-1, stattic, and siRAGE abolished this effect (Figure 7(a)). The determination of the red/green ratio also showed that the decrease of this ratio by CML-BSA was reversed by treatment with Mdivi-1, stattic, and siRAGE (Figure 7(b)).

### 3.4. RAGE-Mediated Activation of JAK2/STAT3 Axis Regulates Vascular Remodeling and Mitochondrial Dynamics of VSMCs in Vivo

The mouse model of type 2 diabetes was created to investigate the effects of Mdivi-1, stattic, and RAGE on mitochondrial dynamics and vascular remodeling in vivo. Then, the vascular tissues were taken and subjected to the Oil red O staining. As shown in Figure 8(a), the results showed the increased presence of lipids in the tissues from diabetic animals compared to normal animals. Compared to diabetic animals, treatments with Mdivi-1, stattic and RAGE inhibited the lipid accumulation observed in the diabetic model (Figure 8(a)). In addition, HE staining showed disorganization of vascular tissue relative to tissues collected from normal animals (Figure 8(b)). In addition, the tissue disorganization observed in diabetic animals was attenuated by the treatments with Mdivi-1, stattic, and RAGE (Figure 8(b)). Furthermore, the immunofluorescence experiment showed *α*-SMA super expression in the vascular tissue of the diabetic group. This super expression was attenuated by Mdivi-1, stattic, and siRAGE in diabetic animals. The same observations were made concerning the expression of VEGF (Figure 9(a)) and CD31 (Figure 9(b)). These results indicated that RAGE-mediated activation of the JAK2/STAT3 axis regulates vascular remodeling via mitochondrial dynamics of VSMCs in vivo.

## 4. Discussion

Diabetes is a disease affecting a large segment of the population, particularly in developing and developed countries. Patients with diabetes are at risk of developing vascular complications, the treatment of which represents an enormous challenge in clinics. The present study demonstrated that RAGE is a vital modulator in vascular remodeling in the diabetic context and this regulation is the result of the modulation of mitochondrial dynamics by the JAK2/STAT3 signaling pathway. This study, as far as we are aware, is the first to establish the relationship between RAGE-JAK2-STAT3-mitochondrial dynamics-vascular remodeling in the diabetic context.

RAGE is a protein that is part of the AGEs-RAGE axis, which is a key route in glucose metabolism. This metabolic pathway has been implicated in the pathophysiology of a variety of diabetes-related illnesses and vascular problems [12–17]. The AGE-RAGE-DIAPH1 axis, for example, has been linked to insulin resistance in the subcutaneous tissue of obese people [18]. Renal failure and kidney ageing are also influenced by the AGE-RAGE axis [19]. RAGE has been shown to have anti-fibrotic properties through the regulation of autophagy inducing endothelial-mesenchymal transition. The blockade of AGEs/RAGE has also been shown to have protective properties by inhibiting endothelin-1 (ET-1) [20]. Additional studies have indicated that the AGE/RAGE pathway plays an important role in diabetes-mediated vascular calcification [14]. However, we were able to demonstrate that RAGE expression is elevated in cellular and animal models of diabetes and that inhibition of RAGE was followed by inhibition of mitochondrial dynamics. The increased expression of RAGE is consistent with numerous studies [16, 17]. Our study, incorporated with the above-mentioned studies, indicated that RAGE plays a significant role in diabetes-mediated vascular remodeling. The pathways in which RAGE is involved are thus potential therapeutic targets for diabetes-related vascular complications. To this end, it is necessary to explore and elucidate thoroughly the processes and molecular mechanisms involved.

Mitochondrial dynamics are essential in diabetes [21]. Here we have tried to help clarify the mechanism governing this process. Our results showed that ROS production associated with mitochondrial dysfunction fundamentally contributes to the phenotypic change of VSMCs cells, which contributes to vascular remodeling as reflected by the changes in cell multiplication, migration, and invasiveness, as well as the alterations in *α*-SMA, CD31, and VEGF-A levels. The changes in phenotypes observed in this study are characteristic of cardiovascular diseases such as atherosclerosis. This was supported by data from the oil red O staining which showed lipid deposition in the vessels of diabetic animals. This shows that the vascular complications associated with diabetes could lead to atherosclerosis and this partly involves the intervention of mitochondrial dynamics. Our results corroborate the findings of previous researchers who showed that mitochondrial dysfunction is a key player in obesity and hypertension [22]. The mitigation of mitochondrial fission by Mst1 knockout in hyperglycemia-mediated vascular damage was also reported [23] and corroborated our present work. Another researcher has also conveyed that the antidiabetic drug metformin exerts its therapeutic effect by inhibition of mitochondrial fission [24]. Our present work contributes in that it proposes RAGE as a therapeutic target for alleviating mitochondrial dysfunction to prevent or heal vascular complications associated with diabetes. Specifically, a major contribution of our work is the proposal of RAGE-JAK2-STAT3 as a novel therapeutic target that would influence the mitochondrial dynamics and restore normal mitochondrial function and prevent vascular complications in diabetes. To our knowledge, only one study has demonstrated the role of the JAK2-STAT3 pathway in Drp1-dependent mitochondrial fission-induced neuroinflammation [25]. Thus, our work, not only demonstrated this relationship in diabetes-associated vascular complications but also demonstrated the upstream regulation of this axis by RAGE.

TRPM is a protein involved in mitochondrial potential. TRPM channels are considered therapeutic targets in obesity and diabetes, as they interfere with various biological processes and diseases [26–29]. Here we have demonstrated that TRPM was overexpressed in diabetes, thus confirming the dysfunction of mitochondrial dynamics in blood vessels in diabetes. We also discovered that the RAGE-JAK2-STAT3 signaling pathway is involved in the regulation of this protein. Only one TRPM (TRPM7) has been shown to be controlled by the JAK2-STAT3 pathway so far [30]. As a result, our research is the first to show a link between TRPM and the RAGE-JAK2-STAT3 axis. Drp1 is a mitochondrial division-related gene. Its dysregulation revealed mitochondrial malfunction in our research. Increased cell proliferation, invasion, and migration were seen after DRP1 suppression. This finding demonstrates how mitochondrial dysfunction contributes to diabetes, which can result in vascular problems due to phenotypic abnormalities in vascular tissue.

## 5. Conclusion

To sum up, our work reported for the first time the implications of the RAGE-JAK2-STAT3 axis in the regulation of diabetes-associated vascular complications by modulating mitochondrial dynamics responsible for the phenotypic switch of VSMCs in diabetes. These data suggest that in diabetes, RAGE modulates vascular remodeling through mitochondrial dynamics by altering the JAK2/STAT3 axis. The findings could be crucial in gaining a better understanding of diabetes-related vascular remodeling. It also contributes to a better cytopathological understanding of diabetic vascular disease and provides a theoretical foundation for novel targets that aid in the prevention and treatment of diabetes-related cardiovascular problems. The present findings might be useful in developing drugs for diabetes and its related complications.

## Figures and Tables

**Figure 1:** RAGE regulates mitochondrial dynamics and JAK2/STAT3 pathway in diabetes. (a) Western blotting analysis of the protein expression of RAGE, Drp1, p-Drp1, Mfn2, JAK2, p-JAK2, STAT3, and p-STAT3 in different treatment groups. (b) Immunofluorescence staining of TRPM in different treatment groups. The experiments were carried out in triplicate and representative images were presented. *Note.* ns = non-significant, ^*∗*^*p* < 0.05, ^*∗∗*^*p* < 0.01, ^*∗∗∗*^*p* < 0.001 and ^*∗∗∗∗*^*p* < 0.0001 compared to control, ^#^*p* < 0.05, ^##^*p* < 0.01 compared to CML-BSA group.

**Figure 2:** RAGE regulates JAK2/STAT3 pathway in diabetic mice. Western blotting analysis of the protein expression of Drp1, p-Drp1, Mfn2, JAK2, p-JAK2, STAT3, and p-STAT3 in different treatment groups. The experiments were carried in triplicate and representative images were presented. *Note.* ns = non-significant, ^*∗∗*^*p* < 0.01, ^*∗∗∗*^*p* < 0.001 and ^*∗∗∗∗*^*p* < 0.0001 compared to control, ^#^*p* < 0.05, ^##^*p* < 0.01 compared to TD2M group.

**Figure 3:** RAGE-mediated activation of JAK2/STAT3 axis regulates the proliferation of VSMCs. (a) Western blotting analysis of the protein expression of Drp1, p-Drp1, Mfn2, JAK2, p-JAK2, STAT3, and p-STAT3 in different treatment groups. (b) Cell viability of VSMCs in different treatment groups. The experiment was carried out in triplicate and representative images were presented. Note: ns = non-significant, ^*∗∗∗*^*p* < 0.001 and ^*∗∗∗∗*^*p* < 0.0001 compared to control, ^#^*p* < 0.05 compared to CML-BSA group, ^$^*p* < 0.05 compared to CML-BSA + siRAGE group.

**Figure 4:** RAGE-mediated activation of JAK2/STAT3 axis regulates the cell cycle, migration and invasion of VSMCs. (a) Cell cycle analysis of VSMCs in different treatment groups by flow cytometry. (b) Cell migration of VSMCs in different treatment groups determined by wound-healing assay. (c) Cell invasion of VSMCs in different treatment groups determined by matrigel Transwell assay. The experiments were carried out in triplicate and representative images were presented. Note: ns = non-significant, ^*∗∗*^*p* < 0.01, ^*∗∗∗*^*p* < 0.001 and ^*∗∗∗∗*^*p* < 0.0001 compared to control, ^#^*p* < 0.05 compared to CML-BSA group, ^$^*p* < 0.05 compared to CML-BSA + siRAGE group.

**Figure 5:** RAGE-mediated activation of JAK2/STAT3 axis regulates ROS and vascular remodeling of VSMCs. (a) ROS analysis of VSMCs in different treatment groups by flow cytometry. (b) Western blot analysis of vascular remodeling-related proteins (*α*-SMA, CD31, VEGF-A) in different treatment groups. The experiments were carried out in triplicate and representative images were presented. *Note.* ns = non-significant, ^*∗∗*^*p* < 0.01, ^*∗∗∗*^*p* < 0.001 and ^*∗∗∗∗*^*p* < 0.0001 compared to control, ^#^*p* < 0.05 compared to CML-BSA group, ^$^*p* < 0.05 compared to CML-BSA + siRAGE group.

**Figure 6:** RAGE-mediated activation of JAK2/STAT3 axis regulates TRPM in VSMCs. The expression of TRPM in different groups was determined by immunofluorescence. The experiments were carried out in triplicate and representative images were presented.

**Figure 7:** RAGE-mediated activation of JAK2/STAT3 axis regulates the depolarization of mitochondrial membrane potential in VSMCs. (a) The depolarization of MMP was detected by JC-1 staining method (the magnification for the figure is 200×). (b) Ratio of red/green fluorescence intensity expressed as mean ± SD of triplicates. The experiments were carried out in triplicate and representative images were presented.

**Figure 8:** RAGE-mediated activation of JAK2/STAT3 axis regulates vascular remodeling of VSMCs in vivo. (a) Oil red O staining and HE histological analysis of aortas of mice from different treatment groups (the magnification for the figure is 200×). (b) Immunofluorescence analysis of *α*-SMA in aorta sections of mice from different treatment groups. The experiments were carried out in triplicate and representative images were presented. The magnification for the figure is 200×.

**Figure 9:** RAGE-mediated activation of JAK2/STAT3 axis regulates the expression of vascular remodeling markers in VSMCs in vivo. (a) Immunofluorescence analysis of VEGF-A in aorta sections of mice from different treatment groups. (b) Immunofluorescence analysis of CD31 in aorta sections of mice from different treatment groups.

## Data Availability

Data generated or analyzed during this study are included in this submitted manuscript.
